This article has been retracted.

# Correlation Decomposition between TCM Syndrome Types and Calcium and Phosphorus Metabolism in 50 Maintenance Hemodialysis Sufferers

**DOI:** 10.1155/2022/3927989

**Published:** 2022-10-05

**Authors:** Yuanyuan Li

**Affiliations:** Department of Nephrology, Suixi County Hospital, Huaibei 235000, China

## Abstract

Aiming to reveal the relationship between TCM syndrome types and calcium and phosphorus metabolism in maintenance hemodialysis (MHD) sufferers, 50 sufferers diagnosed with MHD who were admitted to Suixi County Hospital in Anhui Province are selected for retrospective decomposition. The data of TCM classification and laboratory indicators of the sufferers are collected. The experimental results indicate that calcium and phosphorus metabolism disorder is common in maintenance hemodialysis patients, especially calcium and phosphorus product and blood phosphorus elevation. The increase of the calcium-phosphorus product is closely related to the mortality and calcification rate of the subcutaneous soft tissue. It can provide a reference for the diagnosis and therapy of abnormal calcium and phosphorus metabolism in sufferers, which is worthy of clinical application.

## 1. Introduction

Maintenance hemodialysis (MHD) treatment refers to the use of hemodialysis or peritoneal dialysis to save the life of patients and is a transitional method to prolong the life of uremic patients [1]. With the increase of various diseases, the number of patients with end-stage renal disease is also increasing year-by-year. Patients undergoing maintenance hemodialysis not only include uremia caused by chronic nephritis, but also uremia caused by diabetes and hypertension. 80% or more of MHD sufferers are accompanied by varying degrees of calcium and phosphorus metabolism disorders [2, 3]. Persistent disturbance of calcium and phosphorus metabolism can lead to secondary hyperparathyroidism, soft tissue and blood vessel calcification, and affect bone metabolism, which is an important factor leading to cardiovascular disease in such sufferers [4]. In clinical therapy, the use of traditional Chinese medicine theory to treat chronic renal failure has obvious advantages, especially for MHD sufferers [5]. It can delay the dialysis interval, reduce the number of dialysis, treat or reduce complications. However, when a sufferer enters hemodialysis, new changes have occurred in the sufferer's TCM syndrome due to the removal of metabolites and water, and the correction of acid, alkali, and electrolytes [6, 7]. However, the current examination on TCM syndrome types and this study analyzed the relationship between calcium and phosphorus metabolism and TCM syndrome types by analyzing the serum calcium, phosphorus, and other indicators of 50 maintenance hemodialysis sufferers.

The rest of the paper is organized as follows: Section 2 discusses related studies, and Section 3 presents the clinical data. The results and analysis are discussed in Section 4, and Section 5 serves as a conclusion, providing the summary.

## 2. Related Work

Hemodialysis is an important method of renal replacement therapy for patients with chronic renal failure. With the continuous development and progress of the hemodialysis technology, the survival period of patients has been prolonged. Chronic complications, mainly cardiovascular and cerebrovascular diseases, have become the main cause of death in hemodialysis patients [11]. At present, there are many comprehensive measures in preventing and treating chronic complications of hemodialysis, such as comparing blood pressure, correcting anemia, treating hyperparathyroidism, reducing blood viscosity, preventing and treating microinflammation and adjusting dialysis procedures. However, patients still often feel fatigue and dizziness, dry mouth, insomnia, anorexia, constipation, night sweat, chest tightness, palpitation, abdominal distension, pruritus, limb spasm, joint spasm, joint pain, and embolism. In mild cases, the quality of life of patients will be affected. While in severe cases, other acute and severe diseases will occur [12]. Therefore, whether Chinese medicine can fully play an active role in preventing and treating chronic complications of hemodialysis patients is a question worthy of consideration for workers engaged in the prevention and treatment of kidney disease by integrating traditional Chinese and Western medicine. With the progress of blood purification technology, uremic patients can rely on dialysis for long-term survival. At the same time, the incidence rate will increase year-by-year. Among them, chronic nephritis, diabetes nephropathy, and hypertensive kidney damage are the main primary diseases causing this disease [13]. The traditional medicine of the motherland believes that the development of human bones is closely related to the kidneys. As early as 2, 000 years ago, the “Huangdi Neijing” put forward the theory that the kidneys govern the bones and generate the marrow [14, 15]. The important role of the kidney in the regulation of calcium and phosphorus metabolism is an important part of the modern medical interpretation of the theory that “kidney dominates the bone.” Such patients also often present with symptoms such as soreness of the waist and knees, and bone pain. To investigate the pathogenesis, it is the evidence of positive, false, and evil [16].

Calcium and phosphorus metabolism disorders are common in MHD. After regular dialysis, hypocalcemia will be enhanced. Although hemodialysis can remove creatinine and blood urea nitrogen with small molecular weights, it is very weak in removing phosphorus and medium-extensive molecular weight parathyroid hormone whose mechanism is similar to that of medium-molecular-weight substances. Studies have shown that 2.5 g of phosphorus can be removed by hemodialysis every 3 weeks, which is far less than the total phosphorus intake per week [17, 18]. The traditional theory of Chinese medicine believes that the kidney can store the essence, contain the Yuan Yin Yuan Yang, and lay the foundation of the Yin and Yang of the five zang-organs and six fu-organs. As the kidney disease goes on for a long time, the kidney element is damaged, and the Yuan Yin or Yuan Yang is damaged. As the final stage of the evolution of the disease symptoms, the kidney's ability to expel turbidity is almost completely lost at this time, while the real evils such as dampness, turbidity, heat, and blood stasis are increasingly rampant. It will lead to the existence of extensive amount of phosphorus and parathyroid hormone in the body of MHD sufferers [19]. Chen et al. indicated that people suffering from this disease are usually in a pathological state of kidney yin and yang deficiency [20]. Chinese medicine believes that blemish can cause blood stasis and reality can also cause blood stasis. From the perspective of modern Chinese medicine, blood phosphorus and parathyroid hormone are all turbid poisons, and turbid poisons are real evils. In addition to damaging the yin and yang qi, it can also lead to or aggravate blood stasis syndrome.

The pathogenesis of the syndrome of “poison” is based on blemish and excess, which is mainly manifested by the lack of the spleen, kidney yin, and kidney yang. Qi is the commander of blood, and when qi moves, blood circulates, and when qi is deficient, blood is stagnant. Li [21] believed that yin and blood coexist and breed each other. It can be observed that qi deficiency, yin blemish, and yang blemish can cause blood stasis, and blood stasis is the most important concurrent syndrome in maintenance hemodialysis sufferers. The syndrome of water-dampness and damp-heat is more common in sufferers with yang deficiency. In sufferers with primary disease of hypertension and diabetes, yin blemish and qi are more common, and many symptoms of secondary hyperparathyroidism and renal bone disease are close to the syndrome of wind-driven wind-dryness. The equipment commonly used in hemodialysis generally includes hemodialysis machine, water therapy system, and dialysate. The hemodialysis machine is an electromechanical integrated device. The dialysate is mainly diluted by the dialysis concentration containing electrolytes and bases, which can maintain the normal electrolyte level of the body and can also provide bases through a higher base concentration to correct acidosis [22, 23]. Calcium and phosphorus metabolism disorders are generally manifested as excessive phosphorus and calcium deficiency, mainly due to the reduction of intestinal absorption of calcium in chronic renal failure, and the resistance of target organs, resulting in decreased renal tubular reabsorption of calcium. Since dialysis can only remove various small molecular solutes, it cannot completely replace the metabolic and endocrine functions of normal kidneys, and some complications of maintenance dialysis may also occur [24, 25].

## 3. Clinical Data

### 3.1. General Information

A retrospective decomposition of 50 sufferers with MHD who are admitted to Suixi County Hospital in Anhui Province from August 2019 to February 2022, including 21 males and 29 females, average age (56.6 + 11.13) years, with average disease duration (52.88 ± 15.96) month. Bicarbonate dialysis was used for all sufferers, the dialyzer is German Jinbao, the calcium concentration of the dialysate is 1.5 mmol/l, and the potassium concentration is 2.0 mmol/l, and the dialysis frequency is 3 times a week for 4 hours each time.

Diagnostic criteria are as follows: (1) those who refer to the diagnostic criteria for chronic renal failure in the ninth edition of practical internal medicine; (2) those who conform to the criterion of Operating Procedures for Blood Purification (2010 Edition) dialysis indications for end-stage renal disease formulated by the Nephrology Branch of the Chinese Medical Association.

Inclusion criteria are as follows: (1) those who meet the above diagnostic criteria; (2) those with hemodialysis time ≥3 months; (3) ESRD sufferers with hemodialysis more than 3 months, regular dialysis not less than twice a week, each dialysis not less than 4 hours; (4) those with blood flow 200–250 ml/min, with unfractionated heparin or low molecular weight heparin for anticoagulation.

Exclusion criteria are as follows: (1) sufferers with severe complications (acute renal failure, severe infection, and multiple organ failure); (2) sufferers with malignant tumors and autoimmune diseases; (3) sufferers with hormones or immunosuppressants; (4) sufferers with peritoneal dialysis; (5) those with severe pulmonary infection; (6) sufferers with advanced tumor, severe heart failure, or recent consideration of kidney transplantation; (7) those with mental disorders, or those who cannot cooperate with the investigator for other reasons.

### 3.2. Examination Procedures

#### 3.2.1. Determination of Laboratory Indicators

5 ml of cubital venous blood is drawn from all the participating testers in the fasting state in the morning, centrifuged at 3 500 r/min for 10 min, the centrifugation radius is 10 cm, and serum is collected for testing. Detection includes predialysis blood calcium (Ca), serum phosphorus (P), calcium and phosphorus product, and parathyroid hormone (PTH).

#### 3.2.2. Criterion of Dialectical Classification

According to the summary of previous retrospective studies, syndrome standards are formulated for this blemish syndrome as follows: spleen and kidney qi deficiency, spleen and kidney yang deficiency, liver and kidney yin deficiency, qi and yin deficiency, and yin and yang deficiency. Besides, the criterion evidences include the following: water damp syndrome, damp-turbid syndrome, damp-heat syndrome, blood stasis syndrome, wind-moving syndrome, and wind-dry syndrome.

#### 3.2.3. Questionnaire Survey

According to 1.2.2 TCM syndrome differentiation, the clinical observation table for the distribution of TCM syndrome types in hemodialysis sufferers is formulated, and all the subjects included in the observation are subjected to a questionnaire survey and a combination of four diagnostic tests to determine the TCM syndrome types. At the same time, two TCM physicians with TCM licenses will conduct syndrome differentiation, respectively. If there is any disagreement, refer to the third TCM physician with a senior professional title.

### 3.3. Statistical Procedures

In this study, all the data are organized, and a corresponding database is established, and all the databases are entered into SPSS 26.0 for data processing. The measurement data is tested for normality, which can be expressed as ($\bar{x}$ ± *s*) and consistent with positive. The data between sets is *F*, and the independent sample *t*-test is used for the data between sets. The paired sample *t*-test is used for the data within the set, and the Mann–Whitney *U* test is used for nonnormality. In addition, Pearson decomposition is performed. When *P* < 0.05, the disparity between the data is considered to be statistically extensive.

## 4. Results and Analysis

### 4.1. Primary Disease of MHD Sufferers

Among them, there are 28 cases (56.0%) of chronic nephritis, 9 cases (18.0%) of diabetic nephropathy, 6 cases (12.0%) of hypertensive renal damage, and 7 cases (13.7%) of other cases. Chronic nephritis is more common, as shown in Figure 1.

### 4.2. Calcium, Phosphorus, and PTH Standards in MHD Sufferers

According to the “2003 KDOQI Clinical Practice Guidelines on Bone Metabolism in Chronic Kidney Disease and Its Diseases”, the target ranges of calcium, phosphorus, calcium-phosphorus product, and parathyroid hormone are met. As shown in Table 1, the compliance rates of the four items in 50 MHD sufferers are 58.0%, 50.0%, 60.0%, and 26.0%.

### 4.3. Distribution Characteristics of TCM Syndrome Types in MHD Sufferers

Among the primary blemish syndromes, spleen-kidney qi blemish syndrome (24.0%) is the most common, followed by liver-kidney yin blemish syndrome (20.0%), as shown in Table 2. Spleen-kidney qi blemish and spleen-kidney yang blemish syndrome combined with damp-turbid syndrome are more common, qi-yin blemish and liver-kidney yin blemish syndrome combined with damp-heat syndrome and blood stasis syndrome are more common, and yin-yang blemish syndrome combined with blood stasis syndrome are more common.  Figure 2 shows the distribution characteristics of TCM syndrome types in MHD sufferers.

### 4.4. Expression of Calcium and Phosphorus Metabolism in MHD Sufferers with Different TCM Syndromes

The average value of *P*, calcium, and phosphorus product in the syndrome of yin and yang blemish is the highest, which is statistically extensive contrast with the other three types (*P* < 0.05). The average value of P in blood stasis syndrome is the highest, which is statistically extensive contrast with the other three types (*P* < 0.05). There is no statistical disparity in Ca levels among the syndrome types, as shown in Table 3.  Table 4 illustrates the expression of calcium, phosphorus, calcium-phosphorus product, and parathyroid hormone in sufferers with positive MHD. ^Δ^*P* < 0.05, ^□^*P* < 0.05, ^*∗*^*P* < 0.05, and ^※^*P* < 0.05 indicate the contrast with spleen-kidney qi blemish syndrome, spleen-kidney yang blemish syndrome, qi-yin blemish syndrome, and liver-kidney yin blemish syndrome, respectively.

### 4.5. Decomposition of the Relationship between Different TCM Syndrome Types and Calcium and Phosphorus Metabolism in MHD Sufferers

The calcium and phosphorus metabolism indexes of all MHD sufferers with different syndromes are collected, and it is found that the calcium and phosphorus metabolism of MHD sufferers is notoriously positively correlated with both the primary blemish syndrome and the criterion syndrome (both *P* < 0.05), as shown in Table 5.  Figure 3 shows the correlation between calcium and phosphorus metabolism and this blemish syndrome, and Figure 4 shows the correlation between calcium and phosphorus metabolism and the criterion pattern.

## 5. Conclusion

In this study, the relationship between TCM syndrome types and calcium and phosphorus metabolism in maintenance hemodialysis sufferers is explored. The experimental results indicate that calcium and phosphorus metabolism disorder is common in maintenance hemodialysis patients, especially calcium and phosphorus product and blood phosphorus elevation. The increase of calcium-phosphorus product is closely related to the mortality and calcification rate of the subcutaneous soft tissue. It can provide a reference for the diagnosis and therapy of abnormal calcium and phosphorus metabolism in sufferers, which is worthy of clinical application. In the future, we will further study how to effectively control the levels of blood calcium, blood phosphorus, and PTH from the perspective of traditional Chinese medicine to improve the quality of life of patients and reduce the occurrence of clinical complications affecting the prognosis of patients.

## Figures and Tables

**Figure 1:** Primary disease of MHD sufferers.

**Figure 2:** Distribution characteristics of TCM syndrome types in MHD sufferers.

**Figure 3:** Correlation between calcium and phosphorus metabolism and this blemish syndrome: (a) Ca and P; (b) CaP and PTH.

**Figure 4:** Correlation between calcium and phosphorus metabolism and criterion pattern: (a) Ca and P; (b) CaP and PTH.

**Table 1:** Calcium and phosphorus and PTH levels in MHD sufferers.

Index	Ca (mmol/1)	P (mmol/1)	CaP (mg^2^/dL^2^)	PTH (pg/ml)
Target range	2.10∼2.37	1.13∼1.78	<55	150∼300
Low criterion *n* (%)	7 (14.0)	2 (4.0)	0 (0.00)	19 (38.00)
Up to criterion *n* (%)	29 (58.00)	25 (50.0)	30 (60.0)	13 (26.0)
High criterion *n* (%)	14 (28.0)	23 (46.0)	20 (40.0)	18 (36.0)

**Table 2:** Distribution characteristics of TCM syndrome types in MHD sufferers (*n* (%)).

Card type	Wet	Dampness	Heat blood	Stasis	Wind	Turbulence
Spleen and kidney qi blemish syndrome (*n* = 12)	3(6.00)	5(10.00)	3(6.00)	1(2.00)	0(0.00)	0(0.00)
Spleen and kidney yang blemish syndrome (*n* = 10)	2(4.00)	4(8.00)	2(4.00)	2(4.00)	0(0.00)	0(0.00)
Qi and Yin blemish syndrome (*n* = 8)	0(0.00)	0(0.00)	3(6.00)	4(8.00)	1(2.00)	0(0.00)
Liver-kidney yin blemish syndrome (*n* = 11)	0(0.00)	3(6.00)	4(8.00)	4(8.00)	0(0.00)	0(0.00)
Yin and Yang blemish syndrome (*n* = 9)	0(0.00)	1(2.00)	2(4.00)	3(6.00)	0(0.00)	0(0.00)
Total (*n* = 509)	5(10.00)	13(26.00)	14(28.00)	17(34.00)	1(2.00)	0(0.00)

**Table 3:** The expression of calcium, phosphorus, calcium-phosphorus product, and parathyroid hormone in MHD sufferers with this blemish syndrome ($\bar{x}$ ± *s*).

Syndromes	Ca (mmol/1)	P (mmol/1)	CaP (mg^2^/dL^2^)	PTH (Pg/ml)
Spleen and kidney qi blemish syndrome	2.32 ± 0.18	1.51 ± 0.47	42.86 ± 14.10	234.94 ± 21.13
Spleen and kidney yang blemish syndrome	2.30 ± 0.23	1.51 ± 0.24	43.13 ± 7.72	264.22 ± 20.47^△^
Qi and yin blemish syndrome	2.33 ± 0.28	1.94 ± 0.49^△□^	54.15 ± 15.18^△□^	291.91 ± 28.04^△□^
Liver and kidney yin blemish syndrome	2.21 ± 0.26	1.97 ± 0.40^△□^	55.42 ± 12.83^△□^	423.54 ± 41.27^△□^^*∗*^
Blemish of yin and yang	2.27 ± 0.35	2.68 ± 1.17^△□^^*∗*^^※^	73.33 ± 26.95^△□^^*∗*^^※^	435.10 ± 37.13^△□^^*∗*^

**Table 4:** expression of calcium, phosphorus, calcium-phosphorus product, and parathyroid hormone in sufferers with positive MHD.

Syndromes	Ca (mmol/1)	P (mmol/1)	CaP (mg^2^/dL^2^)	PTH (Pg/ml)
Wet certificate	2.16 ± 0.17	1.66 ± 0.46	48.15 ± 26.85	329.26 ± 36.53
Wet turbidity	2.28 ± 0.38	1.58 ± 0.36	53.27 ± 15.05	340.19 ± 17.15^△^
Damp heat syndrome	2.31 ± 0.24	1.88 ± 0.52^△□^	56.45 ± 14.69^△^	376.26 ± 24.06^△□^
Blood stasis syndrome	2.35 ± 0.21	2.14 ± 0.17^△□^^*∗*^	59.03 ± 19.85^△□^	378.97 ± 22.43^△□^

**Table 5:** Decomposition of the relationship between different TCM syndrome types and calcium and phosphorus metabolism in MHD sufferers.

Syndromes	Ca		P		CaP		PTH	
	*r*	*P*	*r*	*P*	*r*	*P*	*r*	*P*
This blemish type	0.397	0.017	0.523	<0.001	0.437	<0.001	0.486	<0.001
Criterion positive	0.326	0.025	0.415	0.004	0.429	0.001	0.515	<0.001

## Data Availability

The simulation experiment data used to support the findings of this study are available from the corresponding author upon request.
